The article "A nexus of social capital-based financing and farmers' scale operation, and its environmental impact" was retracted in 2025. Reasons: unreliable results or conclusions; a conflict of interest; concerns about the peer review; concerns about the citations.

# A nexus of social capital-based financing and farmers' scale operation, and its environmental impact

**DOI:** 10.3389/fpsyg.2022.950046

**Published:** 2022-08-01

**Authors:** Zenghui Li, Zhixin Zhang, Ehsan Elahi, Xin Ding, Jiaqi Li

**Affiliations:** School of Economics, Shandong University of Technology, Zibo, China

**Keywords:** social capital, formal financing, informal financing, farmers' scale operation, environmental impact

## Abstract

The study constructs a theoretical model of social capital, farm household financing, and scale operation and their environmental effects, and conducts an empirical test based on data from China Family Panel Studies (CFPS) which is conducted in 2018 using causal mediation analysis. The results showed that farmers who spent more on human interaction have a higher probability of choosing scale operation by renting land, the mechanism of which is that the social capital accumulated by farmers based on human interaction facilitates their access to formal and informal financing, which in turn alleviates the financing constraint of scale operation. In addition, we found that the farmers with low education were more dependent on social capital to obtain informal financing to achieve scale operation. The environmental effects of scale operation found that the farmers significantly reduced the proportion of fertilizer and pesticide use, which could effectively mitigate possible pollution problems caused by excessive fertilizer and pesticide use. These findings confirm that social capital can alleviate the financing constraints of farmers to expand their operation scale through formal and informal financing, which in turn has a positive environmental effect.

## Introduction

Agricultural scale operation is an important agricultural policy in China. The policy is to achieve large-scale production by promoting land transfer among farmers to achieve multiple goals such as increasing farmers' income, improving agricultural production efficiency, and achieving green development in agriculture. In the past, small-scale farmers often used excessive pesticides, plastic films, and chemical fertilizers, which caused serious environmental pollution and threatened the health of citizens (Ju et al., 2016). Therefore, how effectively achieving agricultural scale management will help to alleviate the pollution problem in the process of agricultural production (Elahi et al., 2021b, 2022a,b).

In developing countries, financing is often one of the difficult problems for small-scale to large-scale farmers (Elahi et al., 2018b; Peng et al., 2021b). With the development of marketization, the substitution of capital is becoming stronger and stronger, and the difficulty of financing has become the main obstacle to the large-scale operation of farmers. In 2015, the National Bureau of Statistics conducted a survey and reported that 82% of family farms have financing needs, and 64% of farmers thought that financing is difficult.

For farmers, social capital is an important support for their financing. Previous studies found that the financing role of social capital is reflected in both formal and informal financing. From the perspective of informal financing, informal financing is a financing channel endogenous to civil society networks. Allen et al. (2019) defined informal financing as a credit that obtains information and execution through social connections. Its mechanism is that social capital such as social relationship networks, trust, and norms can reduce information asymmetry, increase trust and help loan covenant enforcement for both parties of informal financing (Deng et al., 2019). From the perspective of formal financing, the formal financial institutions such as banks often pay more attention to the borrower's repayment ability. However, due to the institutional inertia formed by customs, history, and culture in China's rural areas, there is often a high institutional cost for formal organizations to be embedded into the village community. These formal financial institutions often take certain measures to embed into the village, which will inevitably be affected by social capital such as human relations and trust. Therefore, studying the influencing factors and environmental effects of farmers' scale operation from the perspective of social capital and financing will help us to have a deeper understanding of the relationship between agricultural production, pollution, and society (Peng et al., 2021a; Zhang et al., 2022a,b).

Farmers' scale operation decision is affected by many factors, and scholars have studied it from two aspects. The first is the subjective factors from the perspective of family livelihood decision-making, including the status of concurrent employment, the level of social security, and the expected benefits of scale operation. The second is the objective factors based on the flow of factors, including agricultural socialization services, land transfer and the issue of the agricultural land property rights system that affects land transfer, the availability of financing for farmers, and related issues of the rural financial system. In most developing countries, farmers often lack financial support for agricultural production. Scholars also pay attention to the financing problem in farmers' scale management and study it from different perspectives. From the perspective of expanding the scale of land operation, farmers' access to a certain scale of financing in the credit market will increase the probability of their agricultural land transfer and expand the scale of their agricultural land transfer (Hou and Huo, 2016). From the perspective of scale operation performance, although the output level of scale operation farmers subject to financing constraints has not been affected, the financing constraints lead to an increase in production costs, which will inhibit farmers from further expanding their operation scale. At present, scholars have only briefly verified the relationship between farmers' scale operation and financing, and have not further discussed the mechanism of financing into formal and informal financing.

In recent years, some scholars have begun to study the influence of rural households' financing behavior on their entrepreneurship, borrowing welfare effect, and consumer behavior from the perspective of social capital (Lu and Li, 2018). In terms of research methods, scholars mostly use the stepwise regression method or add cross multiplication terms to the regression equation to test the mechanism (Elahi et al., 2019b,c, 2020). However, due to the strong endogeneity of social capital and informal financing, the determination of causality is very important. These methods have great limitations in endogenetic treatment, which makes it difficult to determine the causal relationship. This paper will use the causal mediation analysis method proposed by Imai et al. (2010a) to overcome the above shortcomings.

The rest of the paper proceeds as follows. In Section Theoretical framework and hypotheses, we explain the mechanism of the study, including the impact of social capital on farmers' scale operation, the intermediary role of financing, and the impact of farmers' scale operation on pesticide and fertilizer reduction. In Section Materials and methods, We describe the microscopic survey data we use, measurement strategy and identification strategy. In Sections Results and discussion and Conclusion and policy implications, we present the empirical results and explores the environmental effects. The last section concludes.

## Theoretical framework and hypotheses

### The impact of social capital on farmers' scale operation

Agricultural scale operation requires the flow and reallocation of production factors to achieve the purpose of large-scale and intensive production (Elahi et al., 2021a). The flow of factors cannot be separated from transactions, and social capital is an important influencing factor in reducing transaction costs. Coase (1937) considers transaction costs as “the cost of using the price mechanism”, including the cost of discovering the relevant price and the object of the transaction, determining the path of the transaction, signing the contract, and monitoring and enforcing the contract. It has been shown that social capital such as social networks, trust, and norms have an important impact on reducing transaction costs and enabling transactions in terms of obtaining transaction information, securing contract enforcement, and reducing moral hazard.

Firstly, social capital can reduce the cost of discovering the relevant prices of production factors and searching for trading partners by facilitating farmers' access to trading information. Currently, the digitalization of rural areas is not high and there is a lack of efficient factor flow platforms. Thus, transactions of production factors such as land, technology, and capital still rely on interpersonal information transfer to obtain transaction information. Social networks are important social capital, and the more developed a farmer's social network is, the wider the sources of information, and the better it is for discovering relative prices and potential trading partners. Transferring to the right size of the land is the basis for achieving scale, so farmers need access to a sufficient amount of information on land leased out. The information transfer advantage of social capital not only enhances farmers' information acquisition ability but also enables them to obtain this information at a lower cost, thus helping them to achieve scale operation (Tran et al., 2018a,b).

Secondly, trust is also an important social capital. It can reduce negotiation costs, reduce problems such as moral hazards due to information asymmetry, and facilitate the conclusion of transactional contracts. Trust is a prerequisite for transactions, and Lu et al. (2019) found that social trust increases the implementation of incomplete contracts in transactions involving relationships, reducing transaction costs, and improving economic efficiency. In the land transfer market, for example, when the property rights system of agricultural land is still imperfect and farmers face property rights risks, farmers tend to transfer their land to friends and relatives who have strong trust relationships. In terms of contract selection, when farmers transfer their land to friends and relatives with close ties and a high degree of trust, they tend to choose incomplete contracts such as oral contracts. Oral contracts have lower transaction costs and higher compliance rates than written contracts. The higher the level of trust and the richer the social capital of the farmer, the higher the expected performance rate and the lower the transaction costs of the deal. This will undoubtedly increase farmers' access to key factors of production such as land and capital, and improve their ability to achieve large-scale operations. Based on the above analysis the following hypothesis is proposed:

H1: Social capital has a catalytic effect on farmers' scale operation.

### The intermediary role of financing

#### Informal financing

Agricultural and rural development in China is generally constrained by financial constraints. Farmers are constrained by a lack of effective loan collateral and high transaction costs, making it difficult for them to obtain financing through formal financial institutions. This financial market failure has resulted in farmers being unable to access the capital needed to expand their operation scale, inhibiting their scale operation, creating inefficiencies in the land transfer market (Deininger and Feder, 2001), and forcing farmers to seek informal financing such as private lending.

Farmers' social capital affects their informal finance in two main ways: first, the network of rural acquaintances constitutes a form of social capital for individuals, and mutual financial assistance within this network may form an informal source of finance as an alternative to formal finance. Informal finance lenders often use information from social networks to vet borrowers and price loans, while farmers with rich social connections are often able to pass on valid credit information and therefore have easier and lower-cost access to the loans needed to expand their businesses (Deng et al., 2019). Secondly, the trust generated by social capital facilitates the conclusion of lending contracts (Guiso et al., 2004) and provides the enforcement of lending contracts. In rural communities, most activities are carried out within a circle of acquaintances, so that relationships are repetitive, stable, and have long-term benefits, making farmers inclined to build long-term trust to obtain long-term benefits. A single default on a loan will result in a loss of trust and penalties for the disruption of future relationships. And default also leads to a loss of credibility within the defaulters' circle of acquaintances, which makes lenders tend to lend to socially capital-rich borrowers, as the richer the social capital the borrower tends to face greater costs of default. Liang et al. (2014) empirically studied the relationship between social capital and farmers' financing ability and found that social capital can improve farmers' informal financing ability, and this effect is more significant in less developed areas.

#### Formal financing

Farmers' social capital also has advantages in accessing formal finance. Firstly, personal financial knowledge plays an important role in an individual's access to formal financial resources. In rural areas, interpersonal relationships are an important way for farmers to access knowledge, technology, and information, and farmers with rich social capital and frequent interpersonal contacts tend to have better financial knowledge, which facilitates their access to formal finance such as financial credit. Secondly, good interpersonal relationships can often find suitable guarantors for loans, which will undoubtedly make it easier for farmers to access bank loans (Hu et al., 2022). Based on the above analysis the following hypothesis is proposed:

H2: Part of the contribution of social capital to farmers' scale operation is channeled through the intermediary mechanism of promoting formal and informal finance for farmers.

### Impact of farmers' scale operation on use of pesticide and fertilizer

Farmers' scale operation is often accompanied by the use of better agricultural machinery and more scientific field management. On the one hand, scientific field management will lead to the scientific planning of inputs of polluting agricultural elements such as fertilizers, pesticides, and mulch. Using the survey data of 1,274 family farms, Zhao et al. (2021) found that the expansion of the operation scale does help reduce the application of chemical fertilizers, and for the family farms with their own labor as the main force, the “reduction effect” of the operation scale is more effective. On the other hand, scientific management will lead to a better selection of relatively fewer polluting pesticides and fertilizers. Secondly, mechanized and precise pesticide spraying and fertilizer application can also precisely control the dosage and achieve pesticide and fertilizer reduction in agricultural production. Zheng and Zhang (2022) found that farmers purchasing specialized agricultural outsourcing services can significantly reduce the use of pesticides, and this pesticide reduction effect is more significant for large-scale farmers.

H3: Farmers' operation scale can reduce the use of pesticides and chemical fertilizers.

## Materials and methods

### Causal effects analysis based on a potential outcome framework

This study draws on a causal mediation analysis approach based on a potential outcome framework constructed by Imai et al. (2010a) to make causal inferences about the impact of social capital on farmers' scale operation and the mediating role of financing.

#### Model design

Firstly, according to the potential outcome framework of Rubin (1974), we assumed that there are *n* farmers (*i* = 1, 2, 3,……, *n*) whose social capital status is denoted as T. To simplify the analysis, here the social capital status of farmers is set to T = 1 (treatment group) i.e., having strong social capital and T = 0 having weak social capital two cases.


(1) $$\begin{array}{r} \tau_{i}\equiv scale_{i}\left(1\right)\;-scale_{i}\left(0\right) \end{array}$$

In the real world, we cannot observe the potential outcomes of a farmer with both high and low-level social capital, so we introduce average total effects (ATE) as


(2) $$\begin{array}{r} \bar{\tau }\equiv E\left[scale_{i}\left(1\right)\;-scale_{i}\left(0\right)\right] \end{array}$$

to study the causal effects between social capital and farmers' scale operation from a general perspective. Afterward, we introduced farmer financing status (*finan*) as a mediating variable to investigate the causal mediation mechanism through which farmer social capital status (T) affects financing and thus farmers' scale operation (*scale*) according to the causal mediation analysis method.

Corresponding to two potential values of financing *finan*_*i*_(0) and *finan*_*i*_(1) under the different intensity of social capital status, the potential outcome *scale*_*i*_(*t, finan*_*i*_(*t*)) of farmers' scale operation has four potential outcomes under different values of mediating variable *finan*_*i*_(*t*) and treatment variable T: *scale*_*i*_(1, *finan*_*i*_(1)), *scale*_*i*_(0, *finan*_*i*_(0)), *scale*_*i*_(1, *finan*_*i*_(0)), *scale*_*i*_(0, *finan*_*i*_(1)). Fixing the value of T in *scale*_*i*_ and simply varying the value of *finan*_*i*_(*t*) at different T, the change of *scale*_*i*_ can indicate the mediating effect of conduction through *finan*_*i*_, i.e., the causal mediating effect. Based on the above analysis, the average causal mediation effects (ACME) can be used as


(3) $$\begin{array}{r} \bar{\delta }\left(t\right)\equiv E\left[scale_{i}\left(t,finan_{i}\left(1\right)\right)\;-scale_{i}\left(t,finan_{i}\left(0\right)\right)\right] \end{array}$$

to represent the causal mediating effect transmitted through the mediating variable *finan*. Similarly, after excluding the effect of informal financing, the causal effect of social capital influencing farmers' scale operation can be expressed as


(4) $$\begin{array}{r} \bar{\zeta }\left(t\right)\equiv E\left[scale_{i}\left(1,finan_{i}\left(t\right)\right)\;-scale_{i}\left(0,finan_{i}\left(t\right)\right)\right] \end{array}$$

i.e., average direct effects (ADE). In addition, under the assumption of no interaction between the treatment variable (T) and the mediating variable (finan), there is the following relationship:


$$\begin{array}{l} \bar{\tau }\;=\;\bar{\delta }\;+\;\bar{\zeta } \end{array}$$

#### Assumptions

According to the causal mediating effects model, to estimate ACME and ADE, a set of assumptions, called the sequential ignorability (SI) assumption, needs to be made for the model. By denoting the observed pretreatment confounders of farmer *i* by *X*_*i*_ and m as the value of the mediating variable *finan*, the sequential ignorability assumption can be written as


(5) $$\begin{array}{r} \left\{scale_{i}\left(t^{{}^{\prime }},m\right),finan_{i}\left(t\right)\right\}\;⊥{\;T}_{i}\;|\;X_{i}=x \end{array}$$

(6) $$\begin{array}{r} scale_{i}\left(t^{{}^{\prime }},m\right)\;⊥\;finan_{i}\left(t\right)\;|\;T_{i}=t,\;X_{i}=x \end{array}$$

Equation 5 indicates that after controlling for a set of confounding variables, the distribution of each farmer's social capital status is randomized, independent of the farmer's financing status and the farmer's scale operation status. In this study, the social capital of farm households refers to the trust, interaction, and mutual assistance between farm households and people within the village based on the rural acquaintance society. The scale operation status and financing status of farmers do not have a direct effect on this interaction status. Considering the possible indirect effects, for example, farmers who operate on a large scale may have stronger economic power, or households with borrowing may be those whose own family economic power may be weaker. In turn, social circles tend to expand or contract and thus expand as economic strength expands or contracts. Thus, annual household income, household size and a range of household head characteristics, and household characteristics are controlled for in the covariate *X*_*i*_ to strengthen the plausibility of the hypothesis.

Equation 6 indicates that after controlling for a set of confounding variables and farmers' social capital status, there are no unobservable factors that are simultaneously associated with *scale*_*i*_ and *finan*_*i*_. Many factors affect both variables, such as farmers with risk appetite tend to finance and tend to expand production; farmers with sufficient household savings do not finance while expanding production, or participation in agricultural cooperatives affects both financing and scale of operation. Although a range of individual, household, and village characteristics and obvious confounding factors were controlled for in the *X*_*i*_ variable as much as possible, this assumption was difficult to fully satisfy due to data availability and objective conditions. Therefore, a sensitivity analysis is used later to further measure the extent to which unobserved confounding factors can have an impact on the robustness of the results.

#### Analytical framework

The traditional mediating effects model examines the mediating effects through the following set of equations (Baron and Kenny, 1986).


(7) $$\begin{array}{r} scale_{i}=\alpha_{1}+\beta_{11}T_{i}+\xi_{1}^{T}X_{i}+\varepsilon_{i1} \end{array}$$

(8) $$\begin{array}{r} finan_{i}=\alpha_{2}+\beta_{21}T_{i}+\xi_{2}^{T}X_{i}+\varepsilon_{i2} \end{array}$$

(9) $$\begin{array}{r} scale_{i}=\alpha_{3}+\beta_{31}T_{i}+\beta_{32}finan_{i}+\xi_{3}^{T}X_{i}+\varepsilon_{i3} \end{array}$$

where α denotes the constant term, β denotes the estimated coefficients of the explanatory variables, ξ denotes the estimated coefficients of the covariates, and ε denotes the error term which is assumed to be normally distributed at zero mean value and constant variance (Abid et al., 2018; Elahi et al., 2018a, 2019a). Based on satisfying the sequential ignorability assumption and the assumption of no interaction between the treatment variables and the mediating variables, the coefficient estimates derived from fitting the above equations can be derived as valid estimates of ACME and ADE by the traditional coefficient product method (Imai et al., 2011), but this method cannot be directly applied to non-linear models. The mediating variable (*finan*) in this study is an ordered multivalued variable. Therefore, it is not possible to estimate consistent estimates of ACME and ADE by estimating the above linear equations. Imai et al. (2010b) used the results of non-parametric identification to construct a general method for calculating ACME and ADE, and provided the corresponding R package “mediation”, whose estimation method consisted of the following steps: (i) fit model (8) (9); (ii) generate potential values of mediating variables under different treatment states based on the fitting the model (8); (iii) substitute into the outcome model (9) to find the four potential outcomes mentioned above respectively; (iv) then find the corresponding ACME and ADE based on Equations (1) and (2); and (v) finally calculate the confidence interval based on a bootstrap method based on asymptotic sampling distribution.

### Data sources

The article selects data from the 2018 China Family Panel Studies (CFPS) to reflect the social, economic, and educational changes in China by tracking data at three levels: individual, family, and community. A questionnaire was used, including a household member questionnaire, a household economic questionnaire, an individual self-response questionnaire, and a proxy questionnaire for parents of young children, containing a total of 14,241 household samples and 58,504 individual samples. The data were processed using the following steps: (i) Household members questionnaire, household economic questionnaire, and individual self-answer questionnaire was combined horizontally; (ii) Rural households were filtered out as samples using individual households in the household economic questionnaire; and (iii) Missing values and outliers of related variables were excluded. After the above processing, a final sample of 6,060 households covering 28 provincial administrative regions and a population of 19,163 people was obtained.

### Variable descriptions

The definitions of variables are given in Table 1. Among them, given the special policy context and social customs in China, it is necessary to explain the variables “scale operation” and “social capital”.

**Table 1:** Summary of variables.

**Variables**	**Definitions**	**Mean**	**Standard deviation**
Scale	Scale operation: Whether farmers rent farmland: Yes=1, No=0	0.113	0.317
Socialc	Social capital: The amount of social spending (log)	7.031	2.525
Finanf	Formal financing: Whether there is a bank loan: Yes = 1, No = 0	0.103	0.304
Finaninf	Informal financing: Whether there are friends, relatives, and private loans: Yes = 1, No = 0	0.163	0.370
Gender	Gender of the head of household: Yes = 1, No = 0	0.509	0.500
Age	The actual age of the head of household	49.243	16.475
Marry	Marital status of the head of household: married = 1, other = 0	0.771	0.420
Edu	Number of years of education of the head of household	6.310	4.616
Insur	Whether the head of the household has at least one kind of medical insurance: Yes = 1, No = 0	0.921	0.270
Popsize	The actual number of household members	3.903	2.000
Income	Annual net household income for the year (log)	10.519	1.126
Medical	Cost of household medical expenses (log)	6.909	2.691
Subsidy	Whether received government subsidies: Yes = 1, No = 0	0.602	0.490
Paf	The average cost of pesticides and fertilizers per acre of farmland	0.746	0.219
Internet	Importance of obtaining information from the Internet	2.492	1.605
Socialnetwork	Importance of obtaining information from acquaintances	2.841	1.370

#### Scale operation

Scale operation is a policy term, not a precise economic term in itself. To justify its measurement, two questions need to be clarified: first, how to define “scale”; and second, why do farmers rent land to represent scale operation.

From the perspective of traditional economic theory, “scale” basically consists of two meanings: first, it is defined from the perspective of production, and second, it is defined from the perspective of input quantity of production factors. From the perspective of production, different agricultural products are not homogeneous or similar, and it is difficult to measure the production of different crops by one standard; from the perspective of production factors, agricultural scale operation can be manifested both as the increase of a single production factor input and as the combined effect of multiple production factors. The factors of production in agriculture contain land, labor, capital, etc., and the core of agricultural scale operation is agricultural scale production based on the scale of land. Therefore, this study uses land scale as the measure of “scale”.

There are two important institutional contexts in which we use whether farmers rent land to characterize farmers' scale operation. First, since the 1980s, the household contract responsibility system has been implemented, under which each village distributes land equally to each household within the village. Due to the objective conditions of China's large population and small land area, it is often difficult to achieve large-scale production on these shared lands. Second, in China, rural land is subject to a system of “three rights”, which divides the property rights of land into ownership, contractual rights, and operation rights. The ownership right is owned by the village collective, while the contractual right and operation right are owned by the farmers. Therefore, the majority of land transfers in China are realized by renting land to form scale operations. Therefore, this paper uses whether a farmer rents land as a reasonable measure of whether a farmer operates on a large scale.

#### Social capital

Social capital is a concept with a wide range of meanings in itself, and Zhang argues that social capital is divided into institutional capital and relational capital. There is a strong link between the concepts of institutional and relational capital, which exist in a mutually reinforcing and interdependent relationship (Lu and Li, 2008). This paper investigates how social capital, which is formed by blood and geopolitical ties in rural acquaintance societies, affects farm household financing and, consequently, farmers' scale operation. Therefore, the social capital referred to in this study is relational capital and does not include institutional social capital such as market and law. Scholars often measure relational social capital by the breadth, depth, and frequency of interactions with friends and relatives, the depth of clan culture, and other indicators such as the total amount of gift expenditures, the presence or absence of genealogy, and the number of friends and relatives who come to the house to pay respects at Chinese New Year. In this paper, social capital is measured by farmers' amount of social spending based on data availability.

## Results and discussion

### Causal mediation analysis of informal and formal financing

Equations (8) and (9) were first fitted and the results are given in Table 2. In particular, the given findings in columns 1 and 2 are the results of the regression with informal finance as the mediating variable and are denoted as Model 1. The given findings in columns 3 and 4 are the results of the regression with formal finance as the mediating variable and are denoted as Model 2. From the data given in columns 1 and 3, it can be seen that the estimated coefficients of social capital are all significantly positive at the 1% level, which indicates that social capital constructed based on human interaction is conducive to farmers' access to informal financing from friends and relatives or private financial institutions, and likewise to formal financing from banks and other financial institutions. The estimated coefficients of both informal financing and social capital in column 2 are significantly positive at the 1% level or higher, and the estimated coefficients of both formal financing and social capital in column 4 are also significantly positive at the 1% level or higher. The above results suggest that farmers with more social capital, who obtained more informal and formal financing, transferred more land to achieve large-scale operations. This provides the basic correlation evidence to verify the intermediation mechanism in the later section.

**Table 2:** Evidence for the relevance of the mediation effect of social capital-based financing for scale operation.

**Variables**	**Model 1**		**Model 2**	
	**(1)**	**(2)**	**(3)**	**(4)**
	**Finaninf**	**Scale**	**Finanf**	**Scale**
Finaninf		0.315***		
		(0.0549)		
Finanf				0.197***
				(0.0670)
Socialc	0.0411***	0.0482***	0.0423***	0.0437***
	(0.00926)	(0.0113)	(0.0114)	(0.0114)
Marry	−0.0899*	0.197***	−0.0382	0.175***
	(0.0497)	(0.0620)	(0.0579)	(0.0622)
Edu	−0.0193***	−0.00427	−0.0170***	−0.00756
	(0.00505)	(0.00572)	(0.00592)	(0.00582)
Medical	0.0594***	0.00416	0.0169*	0.00777
	(0.00827)	(0.00902)	(0.00887)	(0.00899)
Popsize	0.0424***	−0.00615	0.0378***	−0.0112
	(0.0105)	(0.0122)	(0.0124)	(0.0127)
Age	−0.0107***	−0.00735***	−0.0122***	−0.00755***
	(0.00150)	(0.00178)	(0.00175)	(0.00178)
Subsidy	0.0985**	0.000265	0.122**	0.00793
	(0.0431)	(0.0485)	(0.0495)	(0.0484)
Insur	0.0819	−0.0447	−0.136	−0.0409
	(0.0732)	(0.0898)	(0.0909)	(0.0900)
Gender	0.102**	−0.0406	0.0884*	−0.0345
	(0.0395)	(0.0447)	(0.0451)	(0.0446)
Income	−0.070***	0.0636**	0.152***	0.0478*
	(0.0206)	(0.0266)	(0.0271)	(0.0263)
Constant	−1.397***	−2.194***	−2.922***	−2.603***
	(0.138)	(0.170)	(0.300)	(0.296)
Pseudo R^2^	0.0441	0.0835	0.0536	0.0789
Observations	6,060	6,060	6,060	6,060

Standard errors are given in the parentheses. ***, **, and * represent level of significance of parameters at 1, 5, and 10%, respectively.

To further explore the mediating mechanism and its effect, we estimated each average effect of the mediating mechanism in a counterfactual framework using causal mediation analysis, and the results are presented in Table 3. Columns (1) and (2) in Table 3 showed the estimated results of causal mediation analysis for Model 1 and Model 2, respectively. The results showed that when informal financing is used as the mediating variable, the total and direct effects of social capital on farmers' scale operation are significantly positive at the 5% significant level, and the mediating effect is significantly positive at the 1% significant level, and the 95% confidence interval does not contain 0. It indicates that the social capital has a significant promotion effect on farmers' scale operation, and part of the effect is transmitted through the promotion of informal financing, with the intermediation effect accounting for about 11.29% of the total effect. When formal financing is used as the mediating variable, the total effect and direct effect of social capital on farmers' scale operation are significantly positive at the 1% level, the mediating effect is significantly positive at the 5% level, and the 95% confidence interval does not contain 0, which also indicates that social capital has a significant promotion effect on farmers' scale operation, and part of the effect is transmitted through the promotion of informal financing. Through the promotion of informal financing, this part of the mediating effect accounts for about 3.65% of the total effect. These results supported hypotheses 1 and 2. Further analysis revealed that the total effects of both paths are very similar and the mediating effects are significant, but the mediating effects are more significant and account for a larger share of the total effect when informal finance is used as a mediating variable than formal finance.

**Table 3:** Causal mediation analysis of informal and formal financing.

**Average effects**	**Model 1: informal financing**	**Model 2: formal financing**
	**(1)**	**(2)**
ACME ($\bar{\delta }$)	0.0620*** [0.0034,0.0067] (0.000)	0.0021** [0.0005,0.01] (0.006)
ADE ($\bar{\zeta }$)	0.0482** [0.0201,0.1002] (0.002)	0.0526*** [0.0027,0.01] (0.000)
ATE ($\bar{\tau }$)	0.0544** [0.0269,0.2522] (0.002)	0.0547*** [0.0030,0.01] (0.000)
Prop. Mediated	0.1129** [0.0529,0.2500] (0.002)	0.0365** [0.000,0.009] (0.006)
*N*	6,060	6,060

***, **, * denote significant at the 1, 5, and 10% levels, respectively; 95% confidence intervals are in middle brackets; p-values are in small brackets. Results were obtained using Bootstrap with bias-corrected and accelerated (BCa) for 1,000 runs.

### Sensitivity analysis

The causal mediating effect requires adherence to the SI hypothesis, but it is not possible to test for compliance with that hypothesis with the observed data. Sensitivity analysis can yield the extent to which the study violates this hypothesis and the results remain robust. Specifically, there may be some factors such as villagers joining specialized cooperatives that make it easier for farmers to access informal sources of finance and at the same time increase the likelihood of farmers operating at scale. However, it is not possible to control for all confounding factors due to data availability and other reasons. Sensitivity analysis can capture the extent to which the estimates remain robust to the effects of confounding factors.

The results in Table 4 showed that ${\tilde{R}}_{M}^{2}{\tilde{R}}_{Y}^{2}$ is 0.0092 and 0.0087 when ACME equals 0, while columns (1)–(4) in Table 2 showed that the product of the decidable coefficients of the Model 1 and Model 2 is about 0.0032 and 0.0035, respectively. The explanatory power of the unobserved confounders for the mediating and outcome variables is greater than the dozen dependent variables in equations (8) and (9) if they exist to change the established conclusions. Therefore, the measurement results are also robust to a certain degree of violation of the SI assumption.

**Table 4:** Mediation sensitivity analysis for average causal mediation effect.

**Model 1: informal financing**		**Model 2: formal financing**	
ρ at which ACME = 0	0.1	ρ at which ACME = 0	0.1
$R_{M}^{*2}R_{Y}^{*2}$ at which ACME = 0	0.01	$R_{M}^{*2}R_{Y}^{*2}$ at which ACME = 0	0.01
${\tilde{R}}_{M}^{2}{\tilde{R}}_{Y}^{2}$ at which ACME = 0	0.0087	${\tilde{R}}_{M}^{2}{\tilde{R}}_{Y}^{2}$ at which ACME = 0	0.0092

*Represents R square derived from unobserved confounders.

### Heterogeneity

From the above study, we found that the financing role of social capital is mainly reflected in informal financing, and for this reason, it is necessary to further explore the heterogeneity of its effects to provide us with a deeper understanding of the mechanisms at play. For this purpose, we conduct a more in-depth study on the gender and education of the farm household.

#### Gender heterogeneity

In the perception of traditional rural areas, males and females engage in socialization for different purposes. Men are more purposeful in socializing, favoring access to relevant social resources. Women are more inclined to emotional bonding, and thus they believe that male heads of households may be better able to play the role of financing social capital. We estimated the mediating effects separately for female and male household heads, and the regression results are shown in Model 3 of Table 5. The total, direct, and mediating effects of social capital on farmers' scale operation for households headed by men and households headed by women are all significantly positive at 1%. While the total, direct, and mediating effects of social capital on farmers' scale operation for households headed by men were not statistically significantly different from those for households headed by women. Contrary to our expectations, male household heads are not better at converting social capital into informal finance. The possible reason is that our model suffers from some identification problems and our use of favor spending as a variable to measure social capital tends to underestimate the strength of social capital in households headed by women since favor spending tends to be purposeful social interactions.

**Table 5:** Causal mediation analysis of formal financing with different characteristics of the householders.

**Average effects**	**Model 3**		**Model 4**	
	**Female**	**Male**	**High education**	**Low education**
	**(1)**	**(2)**	**(3)**	**(4)**
ACME($\bar{\delta }$)	0.0594*** [0.024, 0.072] (0.000)	0.0646*** [0.035,0.078] (0.000)	0.0433*** [0.023,0.10] (0.000)	0.0784*** [0.046,0.11] (0.000)
ADE ($\bar{\zeta }$)	0.4678*** [0.17, 0.83] (0.000)	0.4960*** [0.17,0.89] (0.000)	0.4816*** [0.10,0.71] (0.000)	0.4833*** [0.14,0.61] (0.000)
ATE ($\bar{\tau }$)	0.5272*** [0.22, 0.91] (0.000)	0.5607*** [0.25,0.97] (0.000)	0.5249*** [0.15,0.86] (0.000)	0.5617*** [0.21,0.71] (0.000)
*N*	6,060	6,060	6,060	6,060

***, **, *denote significance level of parameters at the 1, 5, and 10%, respectively. 95% confidence intervals are given in middle brackets. p-values are given in small brackets. Results were obtained using Bootstrap with bias-corrected and accelerated (BCa) for 1,000 runs.

#### Educational heterogeneity

We simultaneously estimated the mediating effects at different levels of education. We estimated their mediation effects separately using the household head's primary education level as low education and high school education level as high education. As shown in model 4 of Table 4, the total, direct and mediating effects of social capital on farmers' scale operation are significantly positive at the 1% level of significance for the household head regardless of whether the farmer has high or low education. The direct effects are relatively close in both groups, but the estimated mediating effect of 0.0784 in the low-education group exceeds that of 0.0433 in the high-education group, suggesting that low-education households use social capital to obtain informal financing and thus operate at a scale better than the high-education group, but the robustness of this finding is questionable due to the lack of precision of the model estimates and the overlap of their 95% confidence intervals. We also analyzed why it is difficult for household heads with high education to play a role in social capital financing. First, the natural trust brought by high education is itself a kind of social capital that is not effectively identified by the “human expenditure”. Therefore, our identification strategy also underestimated the sample with high education. Second, highly educated farmers tend to have better formal financing ability and do not need informal financing to meet their financial needs.

### Environmental impact of framers' scale operation on use of agrochemicals

In the next step, we estimated the environmental effects of farmers' scale operation by testing hypothesis 3. To do this we constructed a simple regression equation to verify whether scale farmers have lower costs of fertilizer and pesticides per acre.


(10) $$\begin{array}{r} paf_{i}=\alpha_{1}+\beta_{1}scale_{i}+\gamma X_{i}+\varepsilon_{i} \end{array}$$

where denotes the cost of pesticides and fertilizers used by farmers *i* per acre of land, *X*_*i*_ denotes the matrix of control variables, β_1_ and γ denotes the estimated coefficients of individual scalars, and α is the constant term. Since data is truncated, we used the Tobit model for regression and OLS for auxiliary illustration (Table 6). The first row of Table 6 showed that the estimated coefficient of farmers' scale operation is negative at the 5% level of significance, which indicates that the total cost of pesticides and fertilizers per acre for large-scale farmers is significantly lower than that for non-scale farmers, and farmers' scale operation will contribute to the reduction of pesticides and fertilizers. Furthermore, the estimated coefficients of social networks and the internet are insignificant and significant (with negative signs) at 1%, respectively. It is found with the higher importance of the internet as a source of access to news from farmers' daily sources, the fewer farmers use fertilizers and pesticides, while the importance of farmers' access to information from others is not correlated with the reduction of pesticides and fertilizers. The estimated coefficients of education and age are significantly negative. This implies that the use of agrochemicals will be reduced with an increase in age and education level. The given results in columns 1, 2, 3, 4, and 5 of Table 6 showed that there are no significant differences in changes in the model (Tobit or OLS) or whether we controlled the community fixed effects. In a comprehensive view, to alleviate the problem of environmental pollution in agricultural production, on the one hand, we must expand the scale of operation to achieve large-scale production. On the other hand, farmers themselves should have a high level of literacy and be able to effectively obtain information from the internet to have more effective agricultural production techniques.

**Table 6:** Regression results of framers' scale operation on use of pesticide and fertilizer.

**Variables**	**(1)**	**(2)**	**(3)**	**(4)**	**(5)**
	**Tobit**	**Tobit**	**OLS**	**Tobit**	**OLS**
	**Paf**	**Paf**	**Paf**	**Paf**	**Paf**
Scale	−0.0194**	−0.0192**	−0.0210**	−0.0209**	−0.0209**
	(0.00949)	(0.00953)	(0.0089)	(0.0088)	(0.0086)
Internet		−0.0223***	−0.0230***	−0.0238***	−0.0238***
		(0.00704)	(0.0071)	(0.0064)	(0.0066)
Edu		−0.0371***	−0.0367**	−0.0175**	−0.0175*
		(0.0090)	(0.0091)	(0.0086)	(0.0090)
Age		−0.0142***	−0.014***	−0.0116***	−0.0116***
		(0.0030)	(0.0028)	(0.0028)	(0.0029)
Socialnetwork		−0.0225	−0.0211	−0.0146	−0.0146
		(0.0246)	(0.0248)	(0.0225)	(0.0238)
Popsize		−0.0191	−0.0204	−0.0997	−0.0997
		(0.0176)	(0.178)	(0.168)	(0.172)
Constant	0.749***	0.868***	0.866***	0.831***	0.831***
	(0.00368)	(0.0226)	(0.0228)	(0.0523)	(0.0509)
Community fixed effects	No	No	No	Yes	Yes
*R*^2^/Pseudo *R*^2^	0.0017	0.0082	0.0106	0.1923	0.2360
Observations	4,176	4,171	4,176	4,176	4,176

Standard errors are given in the parentheses. ***, **, and * represent level of significance of parameters at 1, 5, and 10%, respectively.

## Conclusion and policy implications

In this study, we examined how farmers' social capital can facilitate financing to achieve scale operation, and specifically, we further explored how this shift in production and operation patterns affects the environment. The main findings of the study are given below.

1. Results found that the social capital significantly promoted farmers' renting land to realize large-scale operations by playing its financing role.

2. Besides, the role of social capital in financing for scale operations is reflected in both formal and informal financing, with the intermediation effect accounting for 3.7 and 11.3%, respectively. The informal financing role of social capital is much larger than that of formal financing.

3. In terms of the characteristics of different householders, householders with low education rely more on informal financing with social capital to achieve scale operation. While the gender of the householders does not show significant heterogeneity. Thus, it can be seen that farmers who tend to be disadvantaged under the market competition mechanism rely more on access to financial resources through human relations.

4. The environmental effects of scale operation found that the farmers' scale operation significantly contributed to the reduction of the use of pesticides and fertilizers, which showed a positive environmental effect. In addition, a reduction in agrochemical use was related to the source of information acquisition, education, and age of the household head. Furthermore, the use of pesticides and fertilizer was reduced with an increase in information, education, and age.

We found the positive environmental effects of social capital's ability to enable farmers to choose environmentally friendly practices through access to formal and informal financing. Recent studies on social capital have focused on examining its role as shared beliefs and goals among the majority of community members and the community's ability to solve the collective action problem (Cao et al., 2022). Nowadays, it is the main issue that how village communities coordinate collective actions to negotiate and confront enterprises on environmental pollution issues, thus producing environmental effects, deserves to be further explored. Solving this issue will not only provide a new perspective for studying the environmental effects of social capital, but also inspire how to reconcile social development and environmental protection in developing countries.

## Data availability statement

The raw data supporting the conclusions of this article will be made available by the authors, without undue reservation.

## Author contributions

ZL, XD, and JL were responsible for the data collection and arrangement of relevant literature, data analysis, and article writing. ZZ and EE supervised the research. EE edited the revised article. All authors contributed to the article and approved the submitted version.

## Funding

The research was supported by the Taishan Young Scholar Program (tsqn202103070), Taishan Scholar Foundation of Shandong Province, China.

## Conflict of interest

The authors declare that the research was conducted in the absence of any commercial or financial relationships that could be construed as a potential conflict of interest.

## Publisher's note

All claims expressed in this article are solely those of the authors and do not necessarily represent those of their affiliated organizations, or those of the publisher, the editors and the reviewers. Any product that may be evaluated in this article, or claim that may be made by its manufacturer, is not guaranteed or endorsed by the publisher.
